# Double-Negative T Cells Attenuate Cisplatin-Induced Acute Kidney Injury via Upregulating IL-10/AT2R Axis

**DOI:** 10.1155/2022/3629373

**Published:** 2022-07-30

**Authors:** Jing Gong, Jingjing Wu, Mingshun Zhang, Weihua Gan

**Affiliations:** ^1^Department of Pediatric Nephrology, The Second Affiliated Hospital of Nanjing Medical University, Nanjing, China; ^2^Department of Respiratory and Critical Care Medicine, The First Affiliated Hospital of Nanjing Medical University, Nanjing, China; ^3^Department of Immunology, Nanjing Medical University, Nanjing, China

## Abstract

**Objective:**

Our previous research showed that TCR+CD4-CD8-double-negative (DN) T cells protect renal epithelial cells from cisplatin-induced acute kidney injury (AKI). Therefore, this study is aimed at investigating the mechanism underlying the effect of DN T cells against Cis-induced AKI.

**Methods:**

HK-2 cells cultured alone or with DN T cells were treated with or without Cis. After treatment, the cell viability and death were analyzed by a CCK-8 kit and flow cytometric assay with Annexin V/PI staining, respectively. The expressions of inflammatory factors in HK-2 and DN T cells were analyzed using qPCR. The expression levels of nephrotoxicity-associated biomarkers (KIM, calbindin, and TIMP-1), Bcl-2, and angiotensin AT2 receptor (AT2R) were determined by Western blot and qPCR.

**Results:**

The administration of cisplatin significantly decreased the cell viability and AT2R expression, and increased cell death, inflammatory factors, and nephrotoxicity-associated biomarkers of HK-2 cells, while these effects were partly attenuated when cocultured with DN T cells. IL-10 expression was significantly increased in DN T cells after coculture, and cisplatin treatment aggravated this elevation. IL-10 supplementation exhibited a similar effect to coculture, whereas anti-IL-10 antibody reversed the effect of coculture on cisplatin-treated HK-2 cells. Finally, PD123319, an AT2R antagonist, also reversed the effect of IL-10 and coculture on the cell viability, death, and the expression of KIM, calbindin, TIMP-1, and Bcl-2 of cisplatin-treated HK-2 cells.

**Conclusions:**

DN T cells protected HK-2 cells from cisplatin-induced injury through IL-10/AT2R axis, which may act as a potential target for the treatment of cisplatin-induced AKI.

## 1. Introduction

Cisplatin is now widely applied for the treatment of multiple cancers, but its major adverse reaction, acute kidney injury (AKI), limits its clinical use and has raised wide concerns [1, 2]. Approximately one-third of patient suffers from AKI after the treatment of cisplatin, and there is no strategy to effectively protect against such nephrotoxicity at present [3]. Hence, elucidating the pathogenesis of AKI induced by cisplatin is significant for developing agents that can attenuate this serious side effect given its widespread use as chemotherapy.

Over the past decades, the common mechanisms of cisplatin-induced AKI have been investigated extensively [4]. Multiple mechanisms are involved in cisplatin-induced nephrotoxicity, including oxidative stress, vascular injury, necrosis, and apoptosis, as well as inflammation. It is widely accepted that cisplatin-induced nephrotoxicity is attributed to platinum accumulation in renal tissue. The accumulation of cisplatin caused the excess production of reactive oxygen species (ROS) and tumor necrosis factor alpha (TNF-*α*) [5, 6], triggering oxidative stress [7], inflammation [8], and apoptotic pathways [9], which in turn to renal tissue damage and resulting in AKI. Recently, various studies emphasized the important role of inflammation in cisplatin-induced AKI. The activation of TNF-*α* and nuclear factor-*κ*B (NF-*κ*B) leads to proinflammatory cytokine production and cell infiltration thereby exacerbating kidney injury [10–12], while the inhibition of these molecules is associated with the improvement of cisplatin-induced AKI [5, 13]. Hence, uncovering the molecular mechanism underlying renal inflammation is an important research area that may lead to a potential therapy for patients with cisplatin-induced AKI.

Inflammatory responses in AKI involve several types of immune cells, including neutrophils, dendritic cells (DCs), macrophages, natural killer cells, and T lymphocytes [14]. DCs play a protective role in cisplatin-induced AKI [15]. Additionally, blocking neutrophil infiltration by the inhibition of the leukotriene B4-leukotriene B4 receptor axis had a protective effect against cisplatin-induced AKI [16]. As a type of T cell possessing tissue-protective, TCR+CD4-CD8-double-negative (DN) T cells are rarely present in the peripheral blood and lymphoid organs but the major T cell population in human and mouse kidneys [17]. Our previous study demonstrated that DN T cells protect kidney proximal tubular epithelial cells (PTECs) from cisplatin-induced AKI *in vitro* and *in vivo* [18]. However, there is very little information on the mechanism underlying the immunoregulatory roles of DN T cells to protect from cisplatin-induced AKI.

The aim of the present study was to perform a preliminary investigation into the effects of DN T cells on cisplatin-induced AKI and the underlying mechanism. Human Kidney 2 (HK-2) cell line was selected as model for receiving cisplatin stimulation in this study since it maintains biochemical properties and activity similar to *in vivo* proximal tubule cells [19].

## 2. Materials and Methods

### 2.1. Chemical Reagents and Antibodies

Cisplatin was purchased from Sigma-Aldrich (St. Louis, MO, USA). Anti-CD4 (RM4-5) APC/FITC/Pacific blue and anti-TCR*β* (H57-597) FITC/BV421, CD45 (30-F11) APC-Cy7/BUV395, anti-CD8*α* (53 ± 6.7) PerCP-Cy5.5/APC-fire750, were purchased from BD Biosciences. Biotin-conjugated anti-CD16/32 (2.4G2) was purchased from BioLegend. Anti-AGTR2, anti-TIMP-1, and anti-KIM-1 antibodies were purchased from R&D systems (MN, USA). Anti-GAPDH and anti-Bcl-2 antibodies were from Santa Cruz Biotechnology, Inc. (CA, USA). Anti-calbindin antibody was purchased from Cell Signaling Technology, Inc. (MA, USA).

### 2.2. Cell Culture

HK-2 cell line was purchased from the Global Bioresource Center and cultured in HyClone™ DMEM/F12 supplemented with 5% FBS (Gibco, USA) at 37°C in a cell culture incubator. HK-2 cells were starved in the culture medium containing 0.5% FBS for 12 h and then administrated with cisplatin of indicated concentrations (20 or 40 *μΜ*) in the medium for 24 h. Then, the cells were subjected to protein extraction or carry out cell proliferation tests.

### 2.3. Coculture of HK-2 and DN T Cells

The coculture experiment was performed as we previously described [18]. In brief, HK-2 cells were plated in the upper chamber of 24-well plates at a density of 1.5 × 10^4^ cells per well and treated with or without cisplatin. DN T cells isolated from PBMCs using double negative T cell isolation kit (130-092-614, Miltenyi, Germany) were added to the lower chamber for cocultured with cisplatin-treated HK-2 cells at a ratio of 10 : 1 for 24 h at 37°C in a cell culture incubator.

### 2.4. CCK-8 Assay

Cell counting kit-8 (CCK-8) assay (Sangon Biotech, China) was applied to determine the cell viability of HK-2 cells. Cells were cultured in a 96-well plate at a density of 5,000 cells per well. 0.5 mg/mL CCK-8 (10 *μ*L) solution was further added to each well, and cells were incubated for another 1 h at 37°C. The optical density was characterized at 450 nm by a microplate reader (Promega, USA).

### 2.5. Annexin V/PI Staining Assay

To detect cell death, Annexin V-FITC and Propidium Iodide (PI) Staining Solution purchased from BD Pharmingen were used in flow cytofluorimetric analyses. The Annexin V corresponding signal provides a very sensitive method for detecting cellular apoptosis, while PI is used to detect necrotic cells. After finishing treatment, HK-2 cells were resuspended in 100 *μ*l per sample of the Annexin V/PI dilution and followed by incubation for 15 min in dark at room temperature. LSRII flow cytometer was used to analyze the indicated cells, and we analyzed the data by the FlowJo software.

### 2.6. Western Blot

The total cell lysates were collected by using precooled radioimmunoprecipitation assay (RIPA) lysis buffer (50 mM Tris–HCl, pH 7.8, 150 mM NaCl, and 1% Triton X-100, pH 7.8) with supplement of protease inhibitors for 30 min on ice, and then, the mixed liquor was centrifuged for 10 min at 14,000 × g. The lysates were subjected to extract protein by sodium dodecylsulfate–polyacrylamide gel electrophoresis (SDS-PAGE) and further transferred to polyvinylidene fluoride membranes (Millipore, USA). All the antibodies were diluted at 1 : 1,000 and then incubated overnight at 4°C. The secondary antibodies, conjugated to HRP, were diluted in TBST buffer (200 mM Tris base, pH 8.0, 1500 mM NaCl, and 0.1% Tween-20) at 1 : 5,000 and incubated for 1 h at room temperature. Enhanced chemiluminescence (ECL) mix was used to visualize the target proteins in a dark room.

### 2.7. Quantitative Reverse-Transcription Polymerase Chain Reaction (RT-qPCR)

The total RNA of HK-2 or DN T cells was extracted by using TRIZOL reagents (Invitrogen, USA) according to the manual instructions. The cDNAs were synthesized by using a PrimeScript™ RT Reagent Kit (Takara Biotechnology, China), and the cDNAs of cells were further subjected to prepare the RT-qPCR samples with target primers and SYBR Green PCR Master Mix (Promega, USA). The samples were optimized for amplification with the following reaction conditions: denaturalization at 95°C for 10 min, 40 cycles at 95°C for 15 s, and 60°C for 1 min. Glyceraldehyde 3- phosphate dehydrogenase (GAPDH) was used for the expression control. Primers used for qPCR are shown in Table 1.

### 2.8. Statistical Analysis

Data were presented as mean ± SEM. Comparisons between groups were determined using one-way analysis of variance (ANOVA) using Prism 7 (GraphPad Software), and *P* < 0.05 indicated a significant difference.

## 3. Results

### 3.1. DN T Cells Attenuated Cisplatin-Induced Injury of HK-2 Cells

To verify the role of DN T cells in cisplatin-induced AKI, CCK-8 assay was conducted in HK-2 cells which were pretreated with cisplatin. The results showed that the addition of DN T cells improved the cell viability of HK-2 cells with either 20 or 40 *μ*M cisplatin, implying that DN T cells might protect HK-2 cells from cisplatin-induced cell death (Figure 1(a)).

To further confirm the protective role of DN T cells in cisplatin-induced cell death, the HK-2 cells were treated with DN T cells and 40 *μ*M cisplatin and then subjected to flow cytometry by AV-FITC and PI staining. Both apoptosis and necrosis of HK-2 cells were enhanced by 40 *μ*M cisplatin, but that was ameliorated by DN T cells, suggesting DN T cells could reduce the apoptosis and necrosis induced by cisplatin (Figures 1(b) and 1(c)). In summary, these results revealed that DN T cells protected HK-2 cells from injury caused by cisplatin via reducing cell death and increasing cell viability.

### 3.2. Cisplatin Promoted IL-10 Expression in DN T Cells

Inflammation is considered to play a vital role in the pathophysiology of cisplatin-induced AKI, and treatment of AKI by regulating the expression of inflammatory factors has been proposed. Therefore, it is necessary to explore whether the addition of DN T cells affects the expression of inflammatory factors. Thus, the expression levels of IL-1*β*, IL-6, TNF-*α*, and IL-10 in HK-2 cells were detected after DN T cell and cisplatin treatment. The expression levels of these inflammatory factors in HK-2 cells were significantly increased after cisplatin treatment compared with the control cells, but their expression levels were decreased upon the coculture with DN T cells, indicating that DN T cells inhibited the inflammatory process of HK-2 cells induced by cisplatin (Figure 2(a)). However, there is no change expression of IL-10 in cisplatin-treated HK-2 cells after the coculture with DN T cells, suggesting that DN T cells did not affect IL-10 expression in HK-2 cells (Figure 2(a)).

Moreover, IL-17A, INF-*γ*, TNF-*α*, and IL-10 within DN T cells were also determined in our study. Upon different treatments, the expressions of IL-17A, INF-*γ*, and TNF-*α* in DN T cells have not changed. Surprisingly, the IL-10 expression in DN T cells was distinctly increased when DN T cells were cocultured with HK-2 cells, while this change was further aggravated by the addition of cisplatin. Meanwhile, the IL-10 expression in DN T cells was also significantly increased after being treated alone by cisplatin, suggesting cisplatin promoted IL-10 secretion in DN T cells (Figure 2(b)). In summary, upon cisplatin administration, the IL-10 expression in DN T cells was increased, and IL-1*β*, IL-6, and TNF-*α* expression levels in HK-2 cells were decreased, implying that DN T cells might protect HK-2 cells from injury caused by cisplatin by affecting the development of inflammation.

### 3.3. Enhanced IL-10 Expression in DN T Cells Reduced HK-2 Cell Injury Induced by Cisplatin

We further investigated whether IL-10 is involved in the protection of HK-2 cells against cisplatin-induced AKI. Consistent with the previous results, coculture with DN T cells could attenuate the cell death induced by cisplatin in HK-2 cells (Figures 3(a)–3(c)). Notably, the addition of IL-10 exerted a similar function to the coculture in cisplatin-treated HK-2 cells, whereas the addition of anti-IL-10 antibody almost neutralized the effects of the coculture on cisplatin-treated HK-2 cells (Figures 3(a)–3(c)).

Furthermore, the expression levels of nephrotoxicity-related markers (KIM, calbindin, and TIMP-1) and the antiapoptosis protein (Bcl-2) were determined by Western blot and qPCR. As shown in Figure 3(d), upon the stimulation of cisplatin, the expression of KIM, calbindin, and TIMP-1 was increased while Bcl-2 expression was reduced in HK-2 cells, confirming the nephrotoxicity of cisplatin for HK-2 cells. The deleterious role of cisplatin was blocked by both the coculture with DN T cells and IL-10 administration. In line with the result of CCK-8 and Annexin V/PI staining assays, the effect of the coculture on the nephrotoxicity-related markers and antiapoptosis protein in HK-2 cells was restored by the addition of anti-IL-10 antibody (Figure 3(d)). These data collectively revealed that the protective function of DN T cells on HK-2 cells under cisplatin is mediated by IL-10.

### 3.4. IL-10-Induced AT2R Expression Protects HK-2 Cells against Cisplatin-Induced AKI

To further uncover the molecular mechanism underlying the protective effect of DN T cells on cisplatin-treated HK-2 cells, the expression of angiotensin AT2 receptor (AT2R, a renoprotective protein that could be regulated by IL-10) at both mRNA and protein levels was determined using Western blot and qPCR. The results showed that the expression of AT2R in HK-2 cells was decreased upon cisplatin treatment (Figures 4(a) and 4(b)). The addition of IL-10 restored the decreased expression of AT2R in cisplatin-treated HK-2 cells (Figures 4(a) and 4(b)). In the meantime, cocultured with DN T cells also increased the expression of AT2R in cisplatin-treated HK-2 cells (Figures 4(a) and 4(b)), suggesting that DN T cells secreted IL-10 resulted in the upregulation of AT2R in cisplatin-treated HK-2 cells. Subsequently, PD123319, a potent antagonist of AT2R, was used to investigate whether AT2R is involved in the process of DN T cells protecting against cisplatin-induced injury in HK-2 cells. CCK-8 assay and flow cytometry showed that the protective effect of DN T cells and IL-10 was both impaired by AT2R inhibition, suggesting that AT2R was involved in the downstream of IL-10 signaling, thereby inhibiting the damage of cisplatin to HK-2 cells (Figures 4(c)–4(e)).

Then, AT2R could influence the expression of nephrotoxicity-associated biomarkers, and antiapoptosis protein was addressed by Western blot assay. Our findings demonstrated that PD123319 effectively increased the expression of KIM, calbindin, and TIMP-1 and reduced the Bcl-2 expression in the cisplatin-treated HK-2 cells added with either DN T cells or IL-10 (Figure 4(f)), suggesting that AT2R suppression could block the effect of DN T cells and IL-10 on these protein expression in cisplatin-treated HK-2 cells. In general, these data indicated that DN T cells attenuated cisplatin-induced AKI by downregulating inflammatory factors of HK-2 cells and possibly upregulating anti-inflammatory factors of HK-2 cells through IL-10/AT2R pathway, which provided evidence for the treatment of cisplatin-induced AKI by inhibiting inflammation.

## 4. Discussion

Emerging evidence from patients and animal models has suggested that inflammation plays a major role in the pathological processes of cisplatin-induced AKI [20]. The complex inflammatory process is coregulated by various types of immune cells and chemokines. Studies have shown that in cisplatin-induced AKI, activated CD4+T cells infiltrate injured kidneys by secreting TNF-*α* [21]. In addition to the pathophysiologic role in AKI, certain immune cells have been proven to inhibit the progression of AKI [14]. CD4+CD25+Foxp3+ regulatory T (Treg) cells exerted the therapeutic potential by facilitating the repair process and reduced proinflammatory cytokine production by other T cell subsets in AKI [22]. Inducing tolerogenic DCs by adenosine 2A receptor agonist could protect the kidney from ischemia-reperfusion injury by suppressing natural killer T cells [23]. All these reports suggested the therapeutic potential of targeting immune cells in AKI. Our recent work has demonstrated that DN T cells, a rare and heterogeneous T lymphocyte subset, function like Tregs by mediating immune-regulatory effect to protect renal epithelial cells from cisplatin-induced AKI [18]. How DN T cells perform the protective function on PTECs remains unclear. The current study, therefore, uncovered the molecular mechanism of DN T cells in attenuating cisplatin-induced AKI. Given that HK-2 cells are a noncancerous and immortalized human epithelial cell line that retain biochemical properties and activity similar to *in vivo* PTECs [19, 24], we selected this cell line for the following studies.

Consistent with our previous findings, coculturing DN T cells with cisplatin-treated HK-2 cells effectively prevented the HK-2 cells from cisplatin-induced injury. The subsequent detection of inflammatory factors revealed that DN T cells could reduce the inflammation of HK-2 cells induced by cisplatin. It has been reported that DN T cells were involved in several diseases by producing inflammatory factors, including IL-17, INF-*γ*, and IL-10 [17, 25]. Therefore, to investigate the inflammation of DN T cells that responds to cisplatin under mono- or coculture conditions, the expression of IL-10, IL-17A, INF-*γ*, and TNF-*α* in DN T cells has been analyzed the meantime. Our data showed that only IL-10 was dramatically influenced in DN T cells under different conditions, which is consistent with the previous finding that renal DN T cells express a high level of IL-10 in the early phase of AKI [17]. These data suggested that DN T cells could decrease IL-1*β*, IL-6, and TNF-*α* levels in cisplatin-treated HK-2 cells by secreting the high levels of IL-10. IL-10 has been proven to protect against renal injury induced by different factors, such as diabetes [26], ischemia-reperfusion [27], and cisplatin [28]. We, therefore, sought to determine whether IL-10 is involved in the protective effect of DN T cells in cisplatin-treated HK-2 cells. As expected, neutralizing IL-10 antibody supplementation abrogated the DN T cells-mediated improvement in cisplatin-induced HK-2 cells, highlighting that IL-10 is a critical mediator of the role of DN T cells in attenuating cisplatin-induced AKI.

Renin-angiotensin system is an important hormonal system involved in regulating renal structure and function, of which abnormal activation triggers the deleterious effects of angiotensin II [29]. As a component of the renin-angiotensin system, angiotensin type 2 (AT 2) receptor (AT2R) is believed to be renoprotective by functionally antagonizing the proinflammatory actions of angiotensin II, rendering to protecting organs from injury, including AKI [30, 31]. Given the close relationship between AT2R and IL-10 has been reported in various research on renal diseases, we wonder whether the renoprotective function of IL-10 is associated with AT2R. In our study, it was found that the expression of AT2R in HK-2 cells was significantly decreased after cisplatin stimulation. Notably, coculture with DN T cells and the addition of IL-10 could both restore AT2R expression in cisplatin-treated HK-2 cells, suggesting that the protective function of IL-10 secreting by DN T cells on HK-2 cells may be mediated by AT2R. Hence, our study used PD123319, an AT2R agonist, to block the function of AT2R and determine whether AT2R is involved in the effect of IL-10 on cisplatin-treated HK-2 cells. As expected, blocking AT2R activation effectively reversed the effect of both DN T cells and IL-10 on the cisplatin-injury of HK-2 cells, which confirmed that AT2R is an important mediator of the protective role of DN T cells in cisplatin-treated HK-2 cells. Since the kidney is only second to the heart in mitochondrial count and oxygen consumption [32], mitochondria damage induced by oxidative stress is another culprit of cisplatin-induced AKI. Except for anti-inflammatory effects, AT2R has been reported to reduce oxidative stress in multiple diseases [33, 34]. Therefore, DN T cells attenuate cisplatin-induced AKI by reducing inflammation and oxidative stress via IL-10/AT2R axis. However, how IL-10 affects the activity of AT2R in cisplatin-treated HK-2 cells remains unknown. Future work uncovering the reason IL-10 derived from DN T cells could further increase AT2R expression to protect HK-2 cells from cisplatin-induced injury will provide new insights into the mechanism of cisplatin-induced AKI.

In conclusion, our findings suggested that DN T cells protected HK-2 cells from cisplatin-induced AKI through IL-10/AT2R axis, which provides important implications for the prevention of cisplatin-induced nephrotoxicity and for the treatment of other renal injury diseases.

## Figures and Tables

**Figure 1:** The effect of DN T cell treatment on the cell injury of cisplatin-induced HK-2 cells. (a) CCK-8 assay and (b, c) flow cytometry of HK-2 cells pretreated with cisplatin and DN T cells; HK-2 cells were treated with different concentrations of cisplatin (20 and 40 *μ*M), and DN T cells were added into the lower chamber. Monoculture of HK-2 cells was included as a control. Statistical significance was defined as ^∗^*P* < 0.05, ^∗∗^*P* < 0.01, and ^∗∗∗^*P* < 0.001.

**Figure 2:** The effect of DN T cell treatment on the inflammatory factors. After being subjected to cisplatin or/and DN T cell coculture. (a) The mRNA levels of IL-1*β*, IL-6, TNF-*α*, and IL-10 in HK-2 cells were detected by RT-qPCR. (b) The mRNA levels of IL-10, IFN-*γ*, IL-17A, and TNF-*α* in DN T cells were detected after being subjected to cisplatin or/and HK-2 cell coculture. Statistical significance was defined as ^∗^*P* < 0.05, ^∗∗^*P* < 0.01, and ^∗∗∗^*P* < 0.001.

**Figure 3:** IL-10 is essential for the prevention of cisplatin-induced AKI. (a) CCK-8 assay and (b, c) flow cytometry of HK-2 cells pretreated with cisplatin, DN T cells, and anti-IL-10 or IL-10; HK-2 cells were pretreated with cisplatin and DN T cells or cisplatin alone, and then, anti-IL-10 or IL-10 was added into the culture. (d) HK-2 cells were treated by the same strategy, and the KIM, calbindin, TIMP-1, and Bcl-2 protein levels of HK-2 were immunoblotted with anti-KIM, anti-calbindin, anti-TIMP-1, and anti-Bcl-2 antibodies; GAPDH was used as an internal control. Statistical significance was defined as ^∗^*P* < 0.05, ^∗∗^*P* < 0.01, and ^∗∗∗^*P* < 0.001.

**Figure 4:** Upregulation of AT2R by adding IL-10 or DN T cells ameliorates cisplatin-induced AKI. The effect of DN T cells or IL-10 on AT2R expression in HK-2 cells pretreated with cisplatin was detected by (a) qPCR and (b) Western blot. Whole-cell lysates from HK-2 cells cotreated with cisplatin and DN T cells or IL-10 were immunoblotted with anti-AT2R antibody. GAPDH was used as a control. (c) CCK-8 assay and (d, e) flow cytometry of HK-2 cells pretreated with cisplatin, PD123319, and DN T cells or IL-10; HK-2 cells were pretreated with cisplatin and DN T cells or IL-10, and then, PD123319 was added into the culture. (d) HK-2 cells were treated by the same strategy, and the KIM, calbindin, TIMP-1, and Bcl-2 protein levels of HK-2 were immunoblotted with anti-KIM, anti-calbindin, anti-TIMP-1, and anti-Bcl-2 antibodies; GAPDH was used as an internal control. Statistical significance was defined as ^∗^*P* < 0.05, ^∗∗^*P* < 0.01, and ^∗∗∗^*P* < 0.001.

**Table 1:** Sequences of PCR primers used in this study.

GAPDH	Forward (5′-3′)	TGTGGGCATCAATGGATTTGG
	Reverse (5′-3′)	ACACCATGTATTCCGGGTCAAT
IL-1*β*	Forward (5′-3′)	TGTGGCAGCTACCTATGTCT
	Reverse (5′-3′)	GGGAACATCACACACTAGCA
IL-6	Forward (5′-3′)	CGGTCCAGTTGCCTTCTCCC
	Reverse (5′-3′)	GAGTGGCTGTCTGTGTGGGG
TNF-*α*	Forward (5′-3′)	CATCTTCTCAAAACTCGAGTGACAA
	Reverse (5′-3′)	TGGGAGTAGATAAGGTACAGCCC
IL-10	Forward (5′-3′)	GCCAAGCCTTGTCTGAGATGATCC
	Reverse (5′-3′)	TTCACATGCGCCTTGATGTCTGG
IFN-*γ*	Forward (5′-3′)	AGCTCTGCATCGTTTTGGGTT
	Reverse (5′-3′)	GTTCCATTATCCGCTACATCTGAA
IL-17A	Forward (5′-3′)	CCTCAAGTTCCACTT
	Reverse (5′-3′)	CACCAGCATCTTCTCCAC
AT2R	Forward (5′-3′)	TAAGCTGATTTATGATAACTGC
	Reverse (5′-3′)	ATATTGAACTGCAGCAACTC

## Data Availability

This manuscript has no associated data.
